The article "Prediction Model of Residual Neural Network for Pathological Confirmed Lymph Node Metastasis of Ovarian Cancer" was published in 2022. Journal: Biomed Res Int.

# Prediction Model of Residual Neural Network for Pathological Confirmed Lymph Node Metastasis of Ovarian Cancer

**DOI:** 10.1155/2022/9646846

**Published:** 2022-10-11

**Authors:** Huanchun Yao, Xinglong Zhang

**Affiliations:** ^1^Department of Cancer, Shengjing Hospital of China Medical University, No. 36, Sanhao Street, Heping District, Shenyang, 110004 Liaoning Province, China; ^2^Department of Hematology, The Fourth Affiliated Hospital of China Medical University, Shenyang, 110032 Liaoning Province, China

## Abstract

**Purpose:**

We want to develop a model for predicting lymph node status based on positron emission computed tomography (PET) images of untreated ovarian cancer patients. We use the feature map formed by wavelet transform and the parameters obtained by image segmentation to build the model. The model is expected to help clinicians and provide additional information about what to do with first-visit patients.

**Materials and Methods:**

Our study included 224 patients with ovarian cancer. We have chosen two main methods to extract information from images. On the one hand, we segmented the image to extract the parameters to evaluate the clustering effect. On the other hand, we used wavelet transform to extract the image's texture information to form the image's feature map. Based on the above two kinds of information, we used residual neural network and support vector machine for modeling.

**Results:**

We established a model to predict lymph node metastasis in patients with primary ovarian cancer using PET images. On the training set, our accuracy was 0.8854, AUC: 0.9472, CI: 0.9098-0.9752, sensitivity was 0.9865, and specificity was 0.7952. On the test set, our accuracy was 0.9104, AUC: 0.9259, CI: 0.8417-0.9889, sensitivity was 0.8125, and specificity was 1.0000.

**Conclusions:**

We used wavelet transform to process the preoperative medical images of ovarian cancer patients, and the residual neural network can effectively predict the lymph node metastasis of ovarian cancer patients, which is undoubted of great significance for patients' staging and treatment options.

## 1. Introduction

Ovarian cancer is one of the most deadly gynecologic malignancies, with the highest incidence in North America and Central and Eastern Europe. According to the recent epidemiological and related cohort studies, the incidence rate of ovarian cancer shows a gradually increasing trend [1]. However, the vast majority of serous carcinomas are not diagnosed until stage III (51%) or IV (29%) because of the lack of symptoms prior to entire abdominal metastases [2], which is very detrimental to the survival of patients. The global overall 5-year survival rate is as low as 30% [3]. Epithelial ovarian cancer is the most crucial pathological type, accounting for more than 90% of all ovarian cancer [4]. Its subtypes include serous, mucinous, endometrioid, and clear cell carcinoma. According to the current research point of view, ovarian cancer, especially epithelial type, often has a high degree of pathological and molecular heterogeneity in the middle and late stages of the tumor [5], which is also an important reason for the different responses to treatment schemes [6]. Although nearly 75% of ovarian cancer patients achieve pathological remission after primary tumor reduction surgery and chemotherapy, 40-60% of ovarian cancer patients will eventually relapse [7], which seriously affects the quality of life and life safety of patients. According to FIGO guidelines, lymph node metastasis directly affects the surgical pathological stage of the tumor [8]. On this basis, lymph node and other organ involvement affects the extent of surgical resection, especially in patients who wish to preserve fertility. After operation, tumor stage will also affect the choice of chemotherapy regimen. Lymphatic invasion is known as a predictor of tumor invasion and affects the survival of patients with ovarian cancer [9]. The lymph node invasion status of patients with ovarian cancer determines the scope of lymph node dissection in tumor reduction surgery and may be related to surgical complications [10]. Researchers have made many efforts to integrate molecular features for accurate prognosis which helps classify patients into risk groups and may provide more personalized treatment. Information on predictors of lymphatic invasion status in patients with ovarian cancer is still lacking, and few molecular prognostic classifiers are available. A study has shown that PET/CT images can partly reflect preoperative lymph node metastasis in patients with ovarian cancer using traditional artificial imaging diagnostic methods. But this approach is not entirely satisfactory [11]. Lymph node metastasis is thought to be associated with the prognosis of ovarian cancer [12].

Traditionally, radiologists subjectively evaluate medical images based on their training and experience to provide an assessment of the diagnostic disease or clinical status. This method produces irresistible instability in image interpretation. Using more automated imaging analysis tools in research or clinical trials can reduce this instability, provide more objective clinical-related information, and seek more beneficial treatment solutions for patients. Radiomics has been introduced as an emerging tool for post-processing images in medical fields such as computed tomography (CT) or magnetic resonance imaging (MR) and developing new quantitative indicators to link qualitative and quantitative imaging data with clinical endpoints to form an interpretable mathematical model [13]. This method does not rely too much on the will of the physician's supervisor, and through computer program, reliability and repeatability are more guaranteed. Texture analysis is a common research method in medical imaging. It requires researchers to extract specific texture features and then explore the relationship between texture features and clinical features. This correlation tends to be relatively simple and restrictive. However, deep learning can form different features for different tasks more flexibly and can also better explain the complex relationship between image features and clinical features. Ovarian cancer is a disease with complex genetic changes, and the heterogeneity of this genome and tumor microenvironment is related to the platinum resistance of patients [14]. For ovarian cancer, a tumor with complex lesions, noninvasive medical image analysis can better distinguish the heterogeneity of related tumors and play a positive role in tumor patients [15].

In the field of medical image, deep learning is one of the most effective methods. Neural network is a kind of model that simulates human brain in order to realize machine learning technology like artificial intelligence. This technique simulates the structure of human neurons to deal with complex problems. In medical laboratory science, researchers use neural networks to count microorganisms [16]. This method can be applied in the environment without human body [17]. In radiology, researchers use deep learning to identify and segment images. A study on acute intracranial haemorrhage showed that using deep learning methods, researchers were able to classify acute intracranial haemorrhage to the level of manual classification [18]. In gastroenterology, researchers use endoscopy to distinguish benign and malignant tumors, which has great significance in the screening of digestive tract tumors [19]. In assisted reproduction, researchers use neural networks to identify sperm [20]. Deep learning has proved its potential in many medical fields.

Researchers have widely used residual neural networks in various feature extraction applications. When the number of layers of deep learning networks is deeper, the target learning ability will theoretically be stronger. However, when the depth of the convolutional neural network reaches a certain level, the classification performance will not be improved, but the network will converge more slowly, and the accuracy rate will decrease. Even if we increase the sample size of the training set to solve the problem of overfitting, the classification performance and accuracy will not be improved. Residual neural network is a solution to this problem. In medicine, residual neural networks are widely used to deal with pathological and medical images.

## 2. Materials and Methods

### 2.1. Study Participants

We reviewed the radiology database of Shengjing Hospital of China Medical University. We identified 270 patients who underwent PET/CT from April 2013 to January 2019. 23 of these patients were excluded due to missing or poor image quality, and 23 were treated before PET or were diagnosed with nonprimary ovarian tumors on subsequent tests. Therefore, a total of 224 patients were included in this study. The inclusion criteria were that the patients did not have endocrine diseases or other primary tumors that could affect ovarian imaging, underwent PET/CT examination, surgery and pathological examination within two weeks at Shengjing Hospital of China Medical University, and were diagnosed with primary ovarian cancer. Previously, we had excluded patients with advanced ovarian cancer with severe invasion of other organs, large necrotic tumors, patients with severe ascites, and patients with the secondary ovarian cancer.

### 2.2. PET/CT

Patients fasted from food and water for more than 6 hours, and their blood glucose was controlled below 7 mmol/L. Patients accepted PET/CT 1 h after injection of 18F-FDG (GE MINItrace II; GE Healthcare, Milwaukee, WI) 0.08-0.16 MCI/kg. PET/CT was performed from the head to the middle of the femur (GE Discovery PET/CT Elite; GE Healthcare, Milwaukee, WI). A 3D PET model was used with a 192∗192 matrix and 2 min/bed position exposure time. Low-dose spiral CT was performed at 120~140 kV and 80 mA. After attenuation correction of CT, PET images were reconstructed using the algorithm of time-of-flight and point-spread-function, including two iterations and 24 subsets.

We used an advantage workstation 4.6 with PET volume computation-assisted reading software (PET VCAR; GE Healthcare, Milwaukee, WI) to measure PET metabolic parameters. Two radiologists with 15 years of experience reviewed the film independently. If no agreement can be reached, we submit the results to a senior physician for a final decision. The software uses an iterative adaptive algorithm to calculate PET parameters, automatically determines the threshold to delineate the tumor edge, and delineates the region of interest (ROI) based on the above information. The radiologist manually corrected the obtained ROI again and determined the final ROI. Ideally, the ROIs should not contain necrotic or cystic components, as shown in Figure 1. In the case of unsatisfactory images, the radiologist delineated the ROIs manually.

### 2.3. Lymph Node Status

We obtained pathological slides from the patients enrolled above. No data were excluded because the diagnosis was not precise. The Pathology Department of Shengjing Hospital of China Medical University diagnosed whether lymph nodes were benign or malignant. Each sample was fixed in 10% buffered formalin solution. Paraffin-embedded and serial sections were made at a thickness of 0.004 mm. Fixed tissues were removed by dehydration in an automatic tissue processor and stained with HE. The samples were first dewaxed in xylene and alcohol. The samples were stained with hematoxylin for 5 minutes and eosin for 3 minutes [21]. Finally, the samples were immersed in alcohol and xylene for dehydration and transparency. The slides were secured with synthetic resin. A senior pathologist diagnosed the pathological sections to determine whether the lymph nodes had metastases from ovarian malignancies.

### 2.4. Image Segmentation

The main processing of images is based on Python. Load the images using the nibabel library [22]. After the image is processed to remove noise, according to the corresponding gray value of each voxel in the 3D ROI, the Gaussian mixture model is used to cluster each voxel. We segmented the PET images according to the clustering results, as shown in Figure 2.

Finally, we calculated the evaluation cluster parameters as modeling parameters. Three features are extracted, which are

1. Calinski-Harabaz index (CHI)

The score S (Formula (1)) is defined as the ratio of between-cluster dispersion to within-cluster dispersion and is calculated by evaluating between-class and within-class variance. The smaller the covariance of the data within categories, the better, and the larger the covariance between categories, the better, in which case CHI will be significant [23]. To sum up, the higher the score, the better the clustering effect.

(1) $$\begin{array}{c} S=\frac{\text{S}{\text{S}}_{B}}{\text{S}{\text{S}}_{W}}\times \frac{N-k}{k-1}. \end{array}$$

Formula (1) is the calculation formula of CHI.

SSB represents the intracluster distance, SSW represents the intercluster distance, the intracluster distance is represented by the distance between the sample point in the cluster and the center point of the cluster, and the intercluster distance is represented by the distance between the sample point and the center point of other clusters. The specific calculation formula is the following formula.

(2) $$\begin{array}{c} \left.\text{CH}=\frac{\left[\sum_{k=1}^{K}\;n_{k}{||c_{k}-c||}^{2}/K-1\right]}{\sum_{k=1}^{K}\;\sum_{i=1}^{n_{k}}{||d_{i}-c_{k}||}^{2}/N-K}\right]. \end{array}$$

Formula (2) is the specific calculation formula of CHI.

(2) Silhouette coefficient

Silhouette coefficient is a way to evaluate the clustering effect [24]. Peter J. Rousseeuw first proposed it in 1986. It combines two factors: cohesion and separation. Based on the same original data, it can be used to evaluate the impact of different algorithms or different operation modes of algorithms on the clustering results (Formula (3)). The average distance between the sample and other sample points in the cluster is defined as the cluster cohesion degree a, and the average distance between the sample and all sample points in the nearest cluster is defined as the cluster separation degree b.

(3) $$\begin{array}{c} s=\frac{b-a}{\max\left(\text{a},\text{b}\right)}. \end{array}$$

Formula (3) is the silhouette coefficient calculation formula for a single sample.

For all samples, the contour coefficient is the average of each sample contour coefficient. The value of this index ranges from -1 to 1. When the degree of separation between clusters B is much larger than the degree of cohesion A, the value of the contour coefficient is approximately 1. In this case, the heterogeneity between clusters is high, but the similarity is poor. Therefore, the closer to 1 the value of this index is, the better the clustering effect.

(3) Davies-Bouldin index

As shown in Formula (4), DBI is an index proposed by David L. Davis and Donald Bouldin to evaluate the advantages and disadvantages of clustering algorithms [25].

(4) $$\begin{array}{c} \text{DB}=\frac{1}{k}\overset{k}{\underset{i=1}{\sum }}\;\underset{i\neq j}{\max}\;\left(\frac{\text{avg}\left(C_{i}\right)+\text{avg}\left(C_{j}\right)}{d_{\text{cen}}\left(C_{i},C_{j}\right)}\right). \end{array}$$

Formula (4) is the DB calculation formula.

The avg (*c*) represents the closeness of clustering clusters, and the formula is as the following formula.

(5) $$\begin{array}{c} \text{avg}\left(C\right)=\frac{2}{\left|C\right|\left(\left|C\right|-1\right)}\underset{1<i<j\leq \left|C\right|}{\sum }\text{ dist}\left(x_{i},x_{j}\right). \end{array}$$

Formula (5) is the avg(*c*) calculation formula.

Calculate the distance of sample points in the cluster, *d* (Formula (6)) represents the distance between the center points of different clusters.

(6) $$\begin{array}{c} d_{\text{cen}}\left(C_{i},C_{j}\right)=\text{dist}\left(u_{i},u_{j}\right). \end{array}$$

Formula (6) is the *d* calculation formula.

### 2.5. Discrete Wavelet Transform

We used 2D discrete wavelet transform to process PET images [26]. First, 1D-DWT is carried out on each image row to obtain the low-frequency component *L* and high-frequency component *H* of the original image in the horizontal direction, and then, 1D-DWT is carried out on each column of the transformed data. The low-frequency component LL in the horizontal and vertical directions, the low-frequency component LH in the horizontal and vertical directions, the low-frequency component HL in the horizontal and vertical directions, and the high-frequency component HH in the horizontal and vertical directions of the original image are obtained. We select three components, LL, LH, and HL, to extract texture information and form the feature map (Figure 3).

ResNet50 is established based on the library TensorFlow. This model is a specific neural network introduced in residual learning for image recognition by He et al., published in 2015 [27]. Due to the use of the global clustering method instead of the connection layer, the model's size is much smaller, which reduces the size of the ResNet model. ResNet's unique feature is looping learning blocks. This means that each layer must be connected to the next, and the distance jumps directly into the layer about two to three hops away. As shown in Figure 4, the model consists of five maximally pooled convolutional layers, followed by a flat layer, a dropout layer, and finally, a single FC layer. 70% of the feature maps are used as training data, and 30% of the feature maps are used as validation data. The training and validation sets' accuracy are the main parameters of supervised model training.

### 2.6. Data Fusion

We obtained features from two different sources, image texture of image segmentation and wavelet transform, and different forms of data, analyzed the predictive ability of each feature for lymph node condition, selected features with strong correlation, and then performed data fusion. On this basis, we established a model again to predict the lymph node condition.

## 3. Result

### 3.1. Clinical Features

The clinical information of the patients is shown in Table 1.

### 3.2. Prediction Model

Our model shows good prediction ability on both training and testing sets. On the training set, our accuracy was 0.8854, AUC: 0.9472, CI: 0.9098-0.9752, sensitivity was 0.9865, and specificity was 0.7952 (Figure 5).

On the test set, our accuracy was 0.9104, AUC: 0.9259, CI: 0.8417-0.9889, sensitivity was 0.8125, and specificity was 1.0000. As shown in Figure 6, there was no overfitting or underfitting of the model.

For the training and test sets, we plotted calibration curves (Figure 7). Our model shows stable and considerable predictive ability in training and test sets.

## 4. Discussion

In this study, we obtained the image data of patients with primary ovarian cancer from the texture feature map formed by wavelet transform and the parameters extracted after tumor segmentation. We use the feature map to train the model, which simplifies the training process of the model and eliminates the interference of nontumor region information to the model. The above two kinds of information were modeled to predict lymph node metastasis in patients with primary ovarian cancer. On the one hand, it provides a reference for radiologists to make a more detailed diagnosis of lymph node metastases in patients with imaging findings that are difficult to detect, and on the other hand, it provides clinicians with additional information at the time of surgery.

Studies have shown that multiple imaging methods have a good effect on detecting lymph node metastasis in primary ovarian cancer [28]. A study has shown that CT or PET/CT can effectively detect pelvic and para-aortic lymph node metastasis in ovarian cancer [11]. However, this approach relies heavily on the personal experience of the radiologist [29].

A study conducted on MR has demonstrated that ovarian cancer is a biologically heterogeneous tumor [30]. In ovarian cancer, this heterogeneity is reflected not only in response to neoadjuvant chemotherapy but also in imaging. From the pathological point of view, uncontrolled tumor growth is accompanied the by uneven distribution of tumor parenchyma and stroma, including blood vessels. This uneven distribution of blood vessels will lead to the formation of tumor subareas with different blood supply and support and the formation of different tumor microenvironments. Under such survival pressure, mutations in different directions were formed in each subregion of the tumor, which further aggravated the uneven distribution of parenchyma and interstitium. In conclusion, the subregion composition of tumors themselves can reflect the heterogeneity of the biological behavior of tumors. In this case, the accuracy of the texture information extracted from the tumor imaging data in reflecting the heterogeneity of the tumor is inferior to the characteristics describing the relationship between the various tumor subregions. Therefore, different from traditional radiomics analysis, we did not choose to directly extract texture information from tumor imaging data or extract texture features of each subregion after segmentation for modeling. After image segmentation, we did not simply use the percentage of the total number of voxels in each subregion to the total number of voxels in ROI as a parameter. However, we extracted three parameters describing the relationship between subregions usually used to evaluate the clustering effect of clustering methods. These three parameters not only consider the differences between subregions but also describe the similarities between subregions, which enables us to have a more detailed description of the subregions within the tumor, that is, the imaging heterogeneity of the tumor.

Texture representation is an important problem in medical image analysis. Image texture can be defined as the spatial relationship of pixel values in an image region. In medical images, we consider texture as a local feature pattern that identifies the image intensity of tissue. Texture also determines the local spectral or frequency content in the image. A local texture change should cause a local spatial frequency change. Texture analysis is of interest in medical imaging because as biological tissues become abnormal during the course of the disease, their underlying texture may also change. In the medical field, wavelet transform is widely used to process signals and medical images, and noise removal is undoubtedly the most common field of its use [31]. At the same time, discrete wavelet transform also shows its unique advantages in the nuclear magnetic examination of the human brain [32]. In this experiment, we selected three wavelet transform subbands containing more information to form the feature map and then used the deep learning method to reflect the lymph node metastasis of ovarian cancer. In fact, with the development of artificial intelligence, computer-aided diagnosis is increasingly used in the field of medicine. According to the global epidemiological situation, there is no doubt that deep learning studies related to COVID-19 are being widely carried out [33]. In addition, the computer-aided diagnosis of breast cancer has been fairly accurate [34]. Due to the number of open source databases, gastrointestinal cancer research is undoubtedly the most widely carried out [35]. Ovarian cancer is the three most common gynecological diseases in the world, especially in the field of medical imaging, including tomography, ultrasonography (US), magnetic resonance imaging (MRI), and other imaging methods. We have made great strides in artificial intelligence technology [36]. Therefore, ResNet50 was also used to investigate the lymph node metastasis of ovarian cancer. Previously, ResNet50 was used in the medical field to detect COVID-19 and was considered good results [37]. In addition, multiple image segmentation methods have been proposed for deep learning of pathology [38]. On the inspection side, a neural network is more effective at identifying microbes [39]. In addition to the simple recognition and segmentation of medical images, deep learning can combine the medical information contained in images with the clinical information of patients to predict the prognosis of patients. A study has shown that combining patient pathology, CT, and genetic information can predict the prognosis of ovarian cancer patients [40]. Of course, manual diagnosis is currently the gold standard of imaging diagnosis. However, computer-aided diagnosis is undoubtedly more sensitive and efficient in finding hidden lesions and exploring the correlation between different medical information of patients. On the one hand, this will effectively reduce the workload of radiologists; on the other hand, it will also quantify the diagnosis.

In previous studies, researcher mainly have adopted two strategies for predicting of lymph node metastasis. One strategy adopts the deep learning method, which divides the tumor's imaging data into different samples according to the scanning level, and uses the whole CT or MRI for learning [41]. Another strategy is to delineate the ROI of the tumor and perform machine learning on the texture features extracted from the ROI [42]. In a variety of different tumors, ROIs covering tumors were used to predict lymph node metastasis. Both texture analysis and deep learning have made good progress. A study has shown that *T*2-weighted magnetic resonance imaging (T2WI) texture features have a high value in predicting preoperative lymph node invasion in rectal cancer [43]. In papillary thyroid carcinoma, MRI can effectively identify lymph node metastasis [44]. An MRI texture analysis based on machine learning has shown that occult lymph node metastases in early oral tongue squamous cell carcinoma can also be effectively identified [45]. And a study using deep learning confirmed that MRI can be used to predict cervical cancer metastasis [46]. The problem with the first strategy is that the tumor is not a normal physiological structure. If the researchers segment the tumor image according to the scan level, they undoubtedly destroys the integrity of the tumor space. Cancer is a heterogeneous disease, both within the tumor and between different patients. So this method of generating datasets is also difficult to standardise. In addition, this method often directly learns the features of the metastatic lymph nodes, ignoring the characteristics of the tumor itself. The problem with the second strategy is that as deep learning techniques mature, traditional machine learning algorithms are no longer the most advanced. In this experiment, after obtaining the 3D ROI, we conducted deep learning on the extracted texture information and the segmented parameters. In addition to obtaining more image information, we pay more attention to the characteristics of the tumor itself, so as to predict the lymph node metastasis. This approach is more clinical.

However, despite the consideration of various problems, there are still several shortcomings in this study. First of all, the data of this study are all from Shengjing Hospital of China Medical University, which has few cases and is not a multicenter study. To ensure the quality of images, it is undoubtedly most important to expand the sample size for radiological model testing. Second, in image segmentation, we use the Gaussian mixture model to segment the image into three subregions. Technically, this segmentation method is beyond criticism. However, whether it is the most accurate segmentation method to reflect the internal subregion of ovarian cancer tumors still needs further experiments to verify the clinical significance of this segmentation method. Typically, imaging subregional changes in patients who develop resistance during chemoradiotherapy, or specific binding probes, are potent answers to this question [47]. A study shows that clustering after hypersegmentation of images can more accurately describe the features of the inner subregions of images [48]. In addition, our modeling only considers the imaging characteristics of patients. For an early warning model, there is no doubt that the inclusion of patients' clinical information can improve the model's accuracy on the premise of ensuring clinical significance. Age, endocrine status, and genetic mutations, common risk factors for ovarian cancer, were not included because data sources limited them. Finally, this study was limited to patients with untreated early-stage ovarian cancer because it was actually to investigate the relationship between tumor heterogeneity and its biological behavior. For patients with treated or advanced ovarian cancer, the heterogeneity on medical imaging has changed and therefore the conclusions of this study are not applicable. In the future, we may consider further prospective experiments to include clinical information to improve the accuracy of the model, follow up on the prognosis of patients, and complete the monitoring of the whole course of ovarian cancer patients.

## 5. Conclusion

In this study, we used PET images of ovarian cancer to segment the images on the one hand and extract feature parameters according to the segmentation results; on the other hand, we used discrete wavelet transform to process the images and extract feature maps. We established a model to predict the presence of lymph node metastasis by the two aspects of information. This method can provide a reference for the treatment of patients, such as surgery and medication, and the prognosis of patients under the noninvasive condition.

## Figures and Tables

**Figure 1:** An example of ROI. (a) is from a 56-year-old patient with primary ovarian cancer who was positive for lymph node metastases. (b) shows the ROI determined according to the above method.

**Figure 2:** An example of segmentation. The same patient is shown in Figure 1. The black area in (a) is the ROI area, and (b) is the ROI area segmented into three different subareas according to our segmentation method and marked with different colors.

**Figure 3:** An example of characteristic map. (a) is a characteristic map of a 62-year-old patient with ovarian cancer who was negative for lymph node metastasis and immunohistochemical results: positive for ER, positive for PR, and negative for P53. (b) is a characteristic map of a 63-year-old patient with ovarian cancer who was negative for lymph node metastases and had immunohistochemical results: positive for ER, positive for PR, and positive for P53. The difference in their feature maps is noticeable.

**Figure 4:** Structure of ResNet50. (a) shows the structure of the Conv block, (b) shows the structure of the Identity block, and (c) shows the structure of ResNet50. In this experiment, we used the classic architecture of ResNet50 without any modification.

**Figure 5:** The sensitivity and specificity curve of the training set.

**Figure 6:** The sensitivity and specificity curve of the test set.

**Figure 7:** Calibration curve. (a) is the calibration curve of the training set, and (b) is the calibration curve of the test set.

**Table 1:** Clinical information of patients in test and training sets.

Age (year)	Training set	Test set
<65	17	7
>65	140	60
Lymph nodes		
Positive	74	32
Negative	83	35
HER-2		
Positive	93	41
Negative	64	26
PR		
Positive	59	23
Negative	98	44
p53		
Positive	101	47
Negative	56	20

HER-2: human epidermal growth factor receptor 2; PR: progesterone receptor. The PR, HER-2, and p53 status of patients was determined by immunohistochemistry.

## Data Availability

The image data used to support the findings of this study are available from the corresponding author upon request.
